The article "Benevolent Leadership and Team Creative Performance: Creative Self-Efficacy and Openness to Experience" was published in 2022. Journal: Front Psychol.

# Benevolent Leadership and Team Creative Performance: Creative Self-Efficacy and Openness to Experience

**DOI:** 10.3389/fpsyg.2021.745991

**Published:** 2022-01-21

**Authors:** Zhichen Xia, Hong Yu, Fan Yang

**Affiliations:** ^1^Normal College, Changshu Institute of Technology, Changshu, China; ^2^School of Education, Soochow University, Suzhou, China

**Keywords:** benevolent leadership, creative self-efficacy, openness to experience, creative team performance, scientific research team

## Abstract

We examine the association between benevolent leadership and team creative performance in scientific research teams. Moreover, the mediating effects of creative self-efficacy and the moderating effects of openness to experience on the relationship were also analyzed. The study sample comprised 251 postgraduates from 58 scientific research teams in Chinese universities. Results revealed that benevolent leadership was positively related to team creative performance, and creative self-efficacy partially mediated this positive relationship. When team personality composition had a high average team level of or a low level of variance on openness to experience, the relationship between creative self-efficacy and team creative performance was stronger. The same situation also occurred as an indirect effect of benevolent leadership on team creative performance through creative self-efficacy. This study suggests that while people may pay focus on benevolent leadership and creative self-efficacy, team personality composition should also be considered in scientific research team practices.

## Introduction

Teamwork appears to be a trend within many organizations, which is used to accomplish complex tasks (Hackman, 2002). The combination of complementary individuals’ knowledge, skills, and other characteristics will result in the optimal achievement of organizational goals, which is the rationale behind structuring work into teams. In higher educational settings, scientific research organizations are increasingly shifting focus from individuals to team-based structures. Scientific research teams have demonstrated the advantage of producing high-impact or frequently cited research (Wuchty et al., 2007). Considering the characteristics of scientific research, scientific research is classified as creativity-generating tasks based on McGrath’s typology (McGrath, 1984), which need to absorb novel ideas, diverse values, and substantial information. Previous theoretical work and empirical studies have identified that team-based structures are essential for team creative performance or productivity (Fay et al., 2015; Salas et al., 2015). Because of these benefits, understanding what stimulates team creative performance at scientific research teams, motivating scientific research teams for better team creative performance has become an important issue.

The article "Benevolent Leadership and Team Creative Performance: Creative Self-Efficacy and Openness to Experience" was published in 2022. Journal: Front Psychol.

Previous studies on team creative performance have explored team input factors such as team membership and team leadership as antecedents in the teamwork model (Mathieu et al., 2008; Brake et al., 2020). Researchers proposed that team leadership is the most dominant influencing factor of organizational innovation (Barsh et al., 2008; Sun et al., 2014; Booms et al., 2017; Lyubovnikova et al., 2017). Benevolent leadership is prevalent and has attracted scholars’ attention in collectivistic cultures (Aycan et al., 2013), which demonstrates individualized and holistic concern for subordinates and their familial well-being. Jin et al. (2016) found that there was benevolent leadership behavior in scientific research teams in Chinese university organizations, and such leadership had a positive effect on team creative performance. However, not all studies have shown uniformly positive effects of benevolent leadership on team outcomes; benevolence may yield neutral or even negative effects (Wu et al., 2012; Chen, 2013; Wang et al., 2013). The inconformity of the effect of benevolent leadership on team creative performance suggest that the leadership-performance relationship may depend on complex intervening mechanisms. We therefore argue that the underlying mediating mechanism of benevolent leadership, which affects team creative performance in scientific research teams, needs to be further explored.

Extant studies have examined the relationship between benevolent leadership and team creative performance using various mediating mechanisms like perceived support, team action processes, and perceived insider status (Chan, 2017; Shen et al., 2017; Li et al., 2018). Although these mediating mechanisms play a significant role in the relationship between benevolent leadership and team creative performance, researchers have ignored the mediating role of creative self-efficacy in the relationship between benevolent leadership and team creative performance. Creative self-efficacy focuses on the domain of creative activity, defined as the self-view “that one has the ability to produce creative outcomes” (Tierney and Farmer, 2002, p. 1138), which is instrumental in predicting team creative performance (Emilia and Mariola, 2018). The findings of previous studies further strengthen this study’s motivation to use creative self-efficacy as a mediating variable. For example, Walumbwa et al. (2018) noted that self-efficacy provided team members with the confidence that they could achieve the expectancy of favorable outcomes. Sarwat and Abbas (2021) demonstrated that creative self-efficacy serves as an important variable for predicting innovative performance. Moreover, benevolent leaders can inspire team members’ hope and foster their courage for tasks, thus boosting team members’ confidence and promoting creative performance (Xu et al., 2018). Creative self-efficacy appears a mediating mechanism that provides an explanation for the influence of benevolent leadership on team creative performance.

The article "Benevolent Leadership and Team Creative Performance: Creative Self-Efficacy and Openness to Experience" was published in 2022. Journal: Front Psychol.

Despite these significant findings, there is a potential area for research to investigate the moderating effect of benevolent leadership on team creative performance. More recently, Li et al. (2018) called future researchers to check the boundary conditions of team personality composition in the benevolent leadership-team performance relationship. Team personality composition may function as an important contextual variable, and may exert top-down influences on the attitudes and behaviors of team members (Prewett et al., 2016). This study responds to this call by using team personality composition of openness to experience as a moderator in the relationship between benevolent leadership and team creative performance. In the Big Five personality model, openness to experience is considered to be the most relevant and noteworthy to creativity (Schilpzand et al., 2011), which refers to an individual’s ability to be flexible and imaginative in his or her work. As aforementioned, benevolent leadership may promote team creative performance through creative self-efficacy. From an interactional perspective, theoretical treatments of the determinants of creative behavior argue that complex interaction between person and situational factors has a major impact on creative behavior (Amabile, 1996). This “can do” motivation, self-efficacy, may interact with the creativity climate of the organization to influence the team creative performance. Hence, we argue that team personality composition of openness to experience as a second-stage moderator in the benevolent leadership-team creative performance linkage.

Previous research examining the effects of team personality composition has operationalized personality in terms of elevation, that is, the team average level of relevant personality traits (Barrick et al., 1998). According to the person-environment fit theory, heterogeneity or homogeneity of some factors results in better or worse team performance (Muchinsky and Monahan, 1987). Given the equal importance of the mean level of and team variance on personality traits in predicting team creative performance, we use the person-environment fit theory to explore the effects of team personality composition on scientific research team creative performance. Hence, this study had two goals: first, testing the influence of benevolent leadership on team creative performance, as well as the mediating role of creative self-efficacy. Second, using person-environment fit theory to investigate different contingency effects that team-mean-level of and team variance on openness to experience have on the relationship between creative self-efficacy and team creative performance. The present study contributes to the literature in at least two ways. First, we examine the role of creative self-efficacy as an underlying mechanism through which benevolent leadership affect team creative performance in higher educational context. Second, this study responds to the scholars who calls for testing the boundary conditions of team personality composition in the benevolent leadership-team performance relationship. We explore the role of team personality composition of openness to experience in the relationship between benevolent leadership and team creative performance, especially examining the heterogeneity or homogeneity of personality in teams on the leadership-outcome relationships at the team level.

The article "Benevolent Leadership and Team Creative Performance: Creative Self-Efficacy and Openness to Experience" was published in 2022. Journal: Front Psychol.

## Theory and Hypotheses

### Benevolent Leadership and Team Creative Performance

Benevolent leadership refers to supervisors who demonstrate concern for their team members’ personal or familial welfare, which is a prevalent management pattern in the Chinese context (Cheng et al., 2002). Benevolent leaders are more likely to provide support and encouragement to their team members, which enhances team members’ motivation and improves their organizational satisfaction (Zhang et al., 2009). In Chinese higher educational settings, benevolent leaders prefer to express individualized concern about their team members’ daily lives and encourage team members when they encounter problems. According to social exchange theory, team members feel obligated to reciprocate and obey leaders when they have a strong sense of support from benevolent leaders (Farh et al., 2006). Team members are more willing to exhibit extra- as well as in-role behaviors, such as expressing their own opinions, motivating critical thinking, and solving problems from different perspectives, which benefit team creative performance (Chen et al., 2014). Empirical research has also reported that benevolent leadership has a positive relationship with team creative performance (Chan, 2017). For example, Markham and Lee (2014) found that family like relationships increased knowledge sharing within and across teams. Given that previous research mainly focused on the effects of benevolent leadership in enterprise settings, the present study extends these results to the scientific research process of Chinese higher educational settings. We therefore formulate the following hypothesis:

**Hypothesis 1:** Benevolent leadership is positively related to team creative performance.

The article "Benevolent Leadership and Team Creative Performance: Creative Self-Efficacy and Openness to Experience" was published in 2022. Journal: Front Psychol.

### The Mediating Role of Creative Self-Efficacy

Creative self-efficacy refers to one’s confidence in their ability to execute and fulfill the specific tasks that related to creativity or innovation. Based on social cognitive theory, creative self-efficacy has a beneficial effect on innovative performance, especially when team members are working on complex, uncertain, and non-routine tasks without standard solutions (Bandura, 1997). Empirical findings also confirm that self-efficacy, especially creative self-efficacy of team members fosters their innovative performance (Tierney and Farmer, 2011; Emilia and Mariola, 2018). For example, Michael et al. (2011) indicated that team members with a high level of self-efficacy could have sufficient positive psychological capital to deal with uncertainties even when faced with difficulties. The effect of creative self-efficacy on creative performance is mainly reflected in the following two aspects: The first aspect, creative self-efficacy affects team members’ efforts in creative activities, and high creative self-efficacy promotes team members’ creative motivation (Andrea et al., 2018). The second aspect, high creative self-efficacy improves team members’ creative process, including meta-cognitive and self-regulative strategies, and ultimately promotes creative performance (Nickerson, 1999). In summary, the reviews cited above suggests that creative self-efficacy may interfere with creative performance. Therefore, we propose that in scientific research teams, creative self-efficacy enhances creative performance.

The core essence of benevolent leadership is to *shi-en* (favor granting) (Chen et al., 2015). Benevolent leadership are likely to plays an important role in offering positive feedback, coaching, and mentoring team members (Wendt et al., 2009), which is effective in increasing team creative performance because it makes team members think that leaders’ behavior represents the affirmation of their work, so that the team members can improve their confidence to overcome difficulties. In scientific research teams, benevolent leaders are likely to help and encourage team members when they encounter problems, which facilitate a supportive atmospheres and cultivate a psychologically safe environment that stimulate team members enthusiastically engage in team tasks, in turn, increases self-efficacy (Emilia and Mariola, 2018). From Tierney and Farmer’s (2002) perspective, supervisors’ support is an important antecedent variable of creative self-efficacy. Thus, creative self-efficacy is proposed to have a mediation effect between benevolent leadership and team creative performance. We therefore formulate the following hypothesis:

**Hypothesis 2:** Creative self-efficacy mediates the relationship between benevolent leadership and team creative performance.

The article "Benevolent Leadership and Team Creative Performance: Creative Self-Efficacy and Openness to Experience" was published in 2022. Journal: Front Psychol.

### Moderating Effect of Openness to Experience

Creative self-efficacy and its impact on innovative performance would be largely dependent on how the team personality composition functions. The configuration of traits among team members should function as an important contextual variable and constraints within which team members work. We focus on the “Big Five” personality dimensions. Of these, openness to experience is critical to predicting creativity-related behavior and laboratory task performance (Feist, 2010), since innovation and creativity are the dominant characteristics of scientific research tasks. Openness to experience refers to the extent to which an individual is open-minded, imaginative, and curious (Costa and McCrae, 1992). Previous studies on the effects of personality mostly focus on individual personality traits, with less attention paid to the effects of team composition in terms of personality. We draw from the person-environment fit theory to explore the contingent effects of the team-mean-level of and team variance on openness to experience. In the following section, we discuss the role of supplementary fit regarding openness to experience.

According to the person-environment fit theory, individual behavior is not only affected by the independent influence of employee and team characteristics, but is also affected by the matching effect of the two (Hunt, 1975). There are two “traditions of research” in the person-environment fit theory framework (Cable and Edwards, 2004, p. 822): complementary and supplementary fit. Complementary fit occurs in teams when a team member possesses the personality that an organization requires, or an organization offers the rewards that a team member wants. Supplementary fit occurs in teams when the team members’ personalities are similar to or they are compatible with one another. In terms of the current study, the most applicable theoretical approach is supplementary fit for the following reasons.

First, teams with a high mean level of openness to experience are composed of adventurous, imaginative, and creative individuals. Thus, teams with a high number of open individuals are more likely to absorb and combine information flexibly, consider a wide range of ideas and perspectives, and seek varied experiences (Park et al., 2018), which has a positive effect on team performance. Thus, teams with a high mean level of openness to experience enhances members’ involvement in the innovation process. Alternatively, teams with a low mean level of openness to experience are composed of self-constrained and obedient individuals. These teams tend to respond to uncertain in a stubborn manner; they may not be proactive in trying to gain unique experiences or sufficiently flexible for constructive discussions. Hence, creative self-efficacy would not benefit and promote team creative performance in these teams.

The article "Benevolent Leadership and Team Creative Performance: Creative Self-Efficacy and Openness to Experience" was published in 2022. Journal: Front Psychol.

Second, examination of a team’s mean levels of openness to experience may not provide a comprehensive view of the relationship between creative self-efficacy and team creative performance. Moreover, variance on personality traits in teams may be as important as the mean level of traits in predicting team outcomes (Bell, 2007). According to the supplementary fit perspective, teams with a low variance on openness to experience are composed of individuals with similar behavior patterns in response to new experiences, situations, or information (Molleman et al., 2004). Similarity in the trait of openness to experience allows team members to cooperate and discuss, which leads to better team creative performance. Teams with a high variance on openness to experience are composed of individuals with different tendencies to respond to unconventional perspectives (Madrid et al., 2014). Highly open individuals are willing to try new things, find alternatives, and absorb different ideas, while less open individuals tend to be inflexible and uncooperative (Bradley et al., 2013). That is, highly open individuals’ flexibility and imagination may be constrained if less open individuals fail to reciprocate in this regard (Prewett et al., 2016). Thus, the positive effect of creative self-efficacy is unlikely in less open individuals.

We therefore formulate the following hypotheses:

**Hypothesis 3a:** The team-mean-level of openness to experience moderates the relationship between creative self-efficacy and team creative performance, such that creative self-efficacy affects team creative performance more positively with higher rather than lower levels of team-mean-level of openness to experience.
**Hypothesis 3b:** Team variance on openness to experience moderates the relationship between creative self-efficacy and team creative performance, such that creative self-efficacy affects team creative performance more positively with lower rather than higher levels of team variance on openness to experience.

### The Moderated Mediation

As mentioned above, benevolent leadership is expected to increase creative self-efficacy, and creative self-efficacy is expected to interact with the team-mean-level of openness to experience or team variance on openness to experience to affect scientific research team creative performance. Thus, we hypothesize the moderated mediation proposed by combining hypotheses 2, 3a, and 3b. The theoretical model and hypotheses are presented in Figure 1.

The article "Benevolent Leadership and Team Creative Performance: Creative Self-Efficacy and Openness to Experience" was published in 2022. Journal: Front Psychol.

**Hypothesis 4a:** The higher the team-mean-level of openness to experience, the stronger the mediating effect of benevolent leadership on team creative performance through creative self-efficacy.
**Hypothesis 4b:** The lower team variance on openness to experience, the stronger the mediating effect of benevolent leadership on team creative performance through creative self-efficacy.

**FIGURE 1:** Hypothesized model.

## Materials and Methods

### Sample and Procedure

Data were collected from team members and their team supervisors from three top universities in Jiangsu Province, China (Nanjing University, Southeast University, and Soochow University). Questionnaires were administered to 307 team members and 71 team supervisors. Team members rated the benevolent leadership, openness to experience, and self-efficacy questionnaires, while team supervisors provided the team creative performance ratings. In total, we obtained useable data from 251 team members and 58 team supervisors after deleting missing and invalid questionnaires. All the response rates were over 80%. The average team size was 19.05 members per team (*SD* = 15.13), the average age of the team members was 25.51 years old (*SD* = 2.21), and 111 were male (44.22%). Most of the team members (68.0%) were master’s degree candidates, while doctoral candidates accounted for 32.0%.

### Measures

#### Benevolent Leadership

Team members rated the benevolence of their team supervisor via eleven items from Cheng et al.’s (2004) paternalistic leadership scale. The sample for the benevolent leadership scale was “My supervisor ordinarily shows a kind concern for my comfort” (1 = “not at all,” 6 = “frequently”). We obtained a Cronbach’s alpha coefficient of 0.94 for the scale ratings in this study. To justify aggregating the individual-level responses to the team level, we calculated the intra-class correlation coefficients ICC(1) (0.36), and the reliability of the group mean values ICC(2) (0.79), which indicated that the variance was attributable to group membership (LeBreton and Senter, 2008), and the reliability of differentiation among groups (Bliese and Halverson, 1998; Bliese, 2000) was high. Further, we also calculated the average inter-rater reliability r_WG(J)_ ($\bar{X}$ = 0.95), indicating that the team members had a high level of agreement in rating the variable (LeBreton et al., 2005). These indexes suggested that it was appropriate to aggregate benevolent leadership to the team level.

The article "Benevolent Leadership and Team Creative Performance: Creative Self-Efficacy and Openness to Experience" was published in 2022. Journal: Front Psychol.

#### Creative Self-Efficacy

Creative self-efficacy was measured using a three-item scale developed by Carmeli and Schaubroeck (2007). Team members rated the creative self-efficacy ranging from 1 (strongly disagree) to 6 (strongly agree). A sample on this scale was “I will be able to overcome many challenges creatively?” Cronbach’s alpha coefficient for creative self-efficacy was 0.88 in this study. The inter-rater reliability r_WG(J)_ ($\bar{X}$ = 0.88) and the intra-class correlation coefficients [ICC(1) = 0.16; ICC(2) = 0.71] were in the acceptable range, which supported the aggregation of creative self-efficacy.

#### Openness to Experience

Openness to experience was assessed using Wang et al.’s (2011) eight-item scale, the Chinese Big Five Personality Inventory Brief Version (CBF-PI-B). The robustness of the scale has been indicated in the Chinese context (Wang et al., 2014; Yu et al., 2014). The sample item was “I have a vivid imagination” (1 = “totally disagree,” 5 = “totally agree”). Cronbach’s alpha coefficient was 0.83 in this study. The inter-rater reliability r_WG(J)_ ($\bar{X}$ = 0.93) and intra-class correlation coefficients [ICC(1) = 0.23; ICC(2) = 0.82] was in the acceptable range, which supported the aggregation of openness to experience.

We operationalized the team-mean-level of openness to experience as the mean of the team members’ openness to experience. The team variance on openness to experience was computed by dividing the standard deviation of openness to experience scores within each team by its group mean as suggested by Tsui and Gutek’s (1999) scale-invariant measure of dispersion.

#### Team Creative Performance

Team supervisors rated team creative performance that was adapted by De Dreu (2002) three-item scale. Sample items were “This is an innovative team,” “Team members often produce new services, methods, or procedures,” and “This team gives little consideration to new and alternative methods and procedures for doing their work” (1 = “strongly disagree,” 5 = “strongly agree”). Cronbach’s alpha coefficient was 0.81 in this study.

#### Control Variables

We controlled for the effects of team size, level, year, and subject. Team size plays an important role in the team process and performance, because the increasing number of team members can increase the psychological distance between individuals (Pearce and Herbik, 2004, p. 297), which determines the number of interpersonal contacts within the team. Team level was measured for inclusion as a control variable (1 = national level; 2 = provincial level; 3 = school level; 4 = general level). In addition, due to differences in team year and team type (1 = Science and engineering; 0 = others [e.g., Social sciences, Arts and humanities]) were controlled for analysis.

The article "Benevolent Leadership and Team Creative Performance: Creative Self-Efficacy and Openness to Experience" was published in 2022. Journal: Front Psychol.

## Results

We conducted a series of confirmatory factor analyses to examine the construct distinctiveness of the four variables at the team level (benevolent leadership, creative self-efficacy, team creative performance, openness to experience). Compared to other models, the four-factor model showed adequate fit indices (χ^2^/*df* = 1.43, *RMR* = 0.01, *RMSEA* = 0.02, *GFI* = 0.98, *IFI* = 0.99, *TLI* = 0.98, *CFI* = 0.99), which supported the construct distinctiveness of the variables.

According to Podsakoff et al.’s (2003) suggestion, we conducted a Harman’s single-factor test of major variables in this study, the accumulated amount of explanatory variance was 63.97%, and the largest factor did not account for a majority of the variance (37.24%). Thus, common method bias was not a serious problem in the present study.

Table 1 presents the means, standard deviations, and correlations among the variables measured in this study. Benevolent leadership had a positive relationship with creative self-efficacy (*r* = 0.29, *p* < 0.05) and team creative performance (*r* = 0.48, *p* < 0.01). Creative self-efficacy was positively related to team creative performance (*r* = 0.40, *p* < 0.01).

**TABLE 1:** Means, standard deviations, and correlations among variables.

Variables	*M*	*SD*	1	2	3	4	5	6	7	8
(1) Team size	19.05	15.13								
(2) Team type	0.62	0.49	0.17							
(3) Team year	2.57	1.01	0.32*	0.37**						
(4) Team level	3.38	1.12	−0.42**	–0.12	–0.26					
(5) Benevolent leadership	3.41	0.61	0.07	–0.18	0.23	–0.07				
(6) Creative self-efficacy	3.27	0.60	0.16	0.09	0.27*	−0.35**	0.29*			
(7) Team creative performance	3.77	0.66	0.01	–0.03	0.15	0.03	0.48**	0.40**		
(8) TMO	3.37	0.28	–0.01	0.03	0.07	–0.07	0.06	–0.14	0.21	
(9) TVO	1.23	0.13	0.09	0.10	0.04	0.05	–0.14	0.01	–0.15	−0.31*

*TMO, team-mean-level of openness to experience; TVO, team variance on openness to experience.*

*p < 0.05, **p < 0.01.

### Test of Mediation

Hierarchical regression analyses were used to test all the hypotheses. As noted in Table 2, benevolent leadership was positively related to team creative performance (β = 0.48, *p* < 0.01), supporting Hypothesis 1. Benevolent leadership was positively related to creative self-efficacy (β = 0.27, *p* < 0.05), creative self-efficacy was positively related to team creative performance (β = 0.35, *p* < 0.05), and benevolent leadership still had a positive effect on team creative performance (β = 0.39, *p* < 0.01) after entering creative self-efficacy. Further, using the SPSS macro program PROCESS proposed by Hayes (2013) to analyze the mediating effect of creative self-efficacy, the indirect effect of benevolent leadership on team creative performance was found to be significant (*b* = 0.08; 95%CI [0.01, 0.22]). These results showed that creative self-efficacy partially mediated the positive effect of benevolent leadership on team creative performance. Hypothesis 2 was therefore supported.

The article "Benevolent Leadership and Team Creative Performance: Creative Self-Efficacy and Openness to Experience" was published in 2022. Journal: Front Psychol.

**TABLE 2:** Moderated regression results for team openness to experience with team creative performance.

Variables	Creative self-efficacy		Team creative performance						
	Model1	Model2	Model1	Model2	Model3	Model4	Model5	Model6	Model7
**Control**									
Team size	–0.03	–0.03	–0.01	–0.01	–0.01	0.02	–0.01	0.01	0.02
Team type	–0.01	0.07	–0.10	0.05	0.03	0.02	0.10	0.03	0.00
Team year	0.20	0.11	0.21	0.04	0.01	–0.02	–0.05	0.01	0.02
Team level	−0.32*	−0.31*	0.07	0.08	0.18	0.22	0.26*	0.19	0.27*
**Main**									
Benevolent leadership		0.27*		0.48**	0.39**	0.36**	0.41**	0.37**	0.39**
Creative self-efficacy					0.35*	0.41**	0.40**	0.35**	0.33*
TMO						0.26*	0.09		
TVO								–0.12	–0.16
**Interaction**									
Creative self-efficacy × TMO							0.33*		
Creative self-efficacy × TVO									−0.28*
*F*	2.51	2.93*	0.50	3.22*	4.19**	4.68***	5.44***	3.74**	4.34**
*R* ^2^	0.16	0.22	0.04	0.24	0.33	0.41	0.47	0.34	0.42
*△R^2^*		0.06*		0.20*	0.09**	0.08***	0.06***	0.01**	0.08**

*n = 58 teams.*

*TMO, team-mean-level of openness to experience; TVO, team variance on openness to experience. All entries are standardized regression coefficients.*

*p < 0.05, **p < 0.01, ***p < 0.001.

### Test of Moderation

Further, when we entered the interaction term of creative self-efficacy and team-mean-level of openness to experience, the team-mean-level of openness to experience was found to moderate the relationship between creative self-efficacy and team creative performance (β = 0.33, *p* < 0.05), supporting H3a. We also conducted simple slope analyses to further explain the moderating effect of the team-mean-level of openness to experience, which were based on one standard deviation above and below the mean (±1 SD) (Aiken and West, 1991). At high levels of openness to experience (+1 SD), creative self-efficacy was positively related to team creative performance (β = 0.65, *p* < 0.001). At low levels of openness to experience (−1 SD), creative self-efficacy was positively related to team creative performance (β = 0.14, *p* > 0.05) but was not significant. This interaction is graphed in Figure 2.

The article "Benevolent Leadership and Team Creative Performance: Creative Self-Efficacy and Openness to Experience" was published in 2022. Journal: Front Psychol.

**FIGURE 2:** Team-mean-level openness—creative self-efficacy interaction for team creative performance.

Similarly, the effect of creative self-efficacy on team creative performance was moderated by team variance on openness to experience (β = −0.28, *p* < 0.05), supporting H3b. Simple slope analyses showed that creative self-efficacy was positively and significantly related to team creative performance only when variance on openness to experience was low (−1 SD) (β = 0.68, *p* < 0.001). When it was high (+1 SD), the relationship was not significant (β = 0.02, *p* > 0.05). Figure 3 demonstrates that the pattern of two-way interaction is as hypothesized.

**FIGURE 3:** Team variance on openness—creative self-efficacy interaction for team creative performance.

### Test of Moderated Mediation

To test the significance of the conditional indirect effects of benevolent leadership on team creative performance through creative self-efficacy at different team-mean-levels of openness to experience and variance on openness to experience, we utilized the SPSS macro program PROCESS designed by Hayes (2013). The team-mean-level of openness to experience moderated the mediating effect of creative self-efficacy significantly (*b* = 0.37, 95%CI [0.15, 0.58]). As shown in Table 3, the indirect effect of benevolent leadership on team creative performance through creative self-efficacy was positive and significant when the team-mean-level of openness to experience was high (*b* = 0.14, 95%CI [0.02, 0.32]), but not significant when the team-mean-level of openness to experience was low (*b* = 0.03, 95%CI [–0.03, 0.16]).

**TABLE 3:** Test of the mediated moderating model.

		Effect	*SE*	CI
Team-mean-level openness to experience	M-SD	0.03	0.05	[–0.03,0.16]
	M	0.09	0.05	[0.01,0.22]
	M + SD	0.14	0.07	[0.02,0.32]
Team variance on openness to experience	M-SD	0.15	0.10	[0.02,0.43]
	M	0.07	0.05	[0.00,0.21]
	M + SD	−0.01	0.06	[–0.14,0.12]

The moderating effect of variance on openness to experience on the mediating effect of creative self-efficacy was significant (*b* = 0.37, 95%CI [0.15, 0.60]). The indirect effect of benevolent leadership on team creative performance through creative self-efficacy was positive and significant when variance on openness to experience was low (*b* = 0.15, 95%CI [0.02, 0.43]), but not significant when team variance on openness to experience was high (*b* = –0.01, 95%CI [–0.14, 0.12]). These results support Hypotheses 4a and 4b.

## Discussion

This study tested the hypotheses related to the relationships between benevolent leadership, creative self-efficacy, and team creative performance, as well as the contingent effects of team personality composition of openness to experience. Compared to existing studies, the contribution of this study is to verify the previous research conclusions in the context of higher education and support that creative self-efficacy plays a significant role in mediating benevolent leadership and team creative performance. At the same time, based on previous studies on team personality, the moderating effect of openness to experience on this relationship is measured from two aspects of homogeneity and heterogeneity, which supports integrating the two perspectives of team personality in existing studies.

The article "Benevolent Leadership and Team Creative Performance: Creative Self-Efficacy and Openness to Experience" was published in 2022. Journal: Front Psychol.

In support of Hypothesis 1, we found that benevolent leadership had a positive relationship with team creative performance, which is consistent with previous literature. Empirical research has suggested that benevolent leadership is beneficial to follower creative performance (Chan and Mak, 2012; Chen et al., 2014). Benevolent leaders establish positive exchange relationships with individual followers by providing personalized care, understanding, and forgiveness, which stimulates followers to obey the leaders’ attitudes and behaviors, and reciprocate with high levels of in- and extra-role behaviors (Li et al., 2018). Our empirical results revealed a positive relationship between benevolent leadership and team creative performance in the context of higher education.

Furthermore, creative self-efficacy mediated the relationship between benevolent leadership and team creative performance, which is in line with Hypothesis 2. Benevolent leaders are likely to create a supportive atmosphere that encourages member participation and consideration of various alternatives (De Dreu and West, 2001). They offer positive feedback by coaching and mentoring team members (Wendt et al., 2009). Team members under benevolent leaders can easily experience positive feelings such as inspired and effective trust, thereby resulting in developing high level of creative self-efficacy. Moreover, the literature supports the idea that creative self-efficacy fosters team creative performance (Gupta and Singh, 2014; Ng and Lucianetti, 2016). This study is consistent with previous findings, in that it shows that creative self-efficacy facilitates team creative performance in scientific research teams. The main reason may be due to the fact that scientific research teams’ creative performance relies on team members synthesizing divergent thinking and mutual exchange perspectives. Through their encouragement and understanding, benevolent leaders can stimulate team member’s creative self-efficacy and create an open climate of debate and negotiation, which, in turn, contributes to team creative performance. Thus, creative self-efficacy was found to play a mediating role in the relationship between benevolent leadership and team creative performance.

The article "Benevolent Leadership and Team Creative Performance: Creative Self-Efficacy and Openness to Experience" was published in 2022. Journal: Front Psychol.

Finally, as proposed in Hypotheses 3a and 3b, the results indicated that when team personality composition had a high average team level of or a low level of variance on openness to experience, the relationship was stronger between creative self-efficacy and team creative performance, as was the indirect effect of benevolent leadership on team creative performance through creative self-efficacy. A high average team level of openness to experience means that team members are highly open to experience within a team. These members are creative, broadminded, and willing to seek alternative ways to solve new problems or new situations they encounter (LePine, 2003). The higher members’ openness to experience, the more they can accept information or knowledge from others, facilitate different ideas to evolve into applicable solutions, and help resolve unique or complex challenges. For example, LePine et al. (2000) found that teams with higher openness were more successful in adapting to changing contexts. In other words, they can strengthen the relationship between creative self-efficacy and team creative performance. Thus, in the current study, team creative performance was greater with a high average team level of openness to experience.

A low level of variance on openness to experience means that team members have either high or low openness to experience. According to the supplementary fit perspective, these team members are similar in terms of their openness to experience. They tend to seek more information and knowledge producing final solutions in response to those demanding substantial cognitive and creative tasks, subsequently boosting team creative performance. In contrast, the positive effects of creative self-efficacy on team creative performance may be constrained by individuals with high and low levels of openness to experience coexistence in a team. Compared with highly open individuals, those with a low level of openness to experience are inclined to be inflexible and display routine behavior, which may impede highly open individuals’ flexibility in cooperation and communication, and in turn, weaken the relationship between creative self-efficacy and team creative performance. The diversity of openness to experience may decrease psychological safety and then impair team creative performance. Thus, in the current study, team creative performance was greater with a low level of variance on openness to experience.

### Theoretical Implications

Our study makes three primary theoretical contributions to the literature. First, using the setting of scientific research teams in Chinese universities, this study complements the empirical evidence of the antecedents of team creative performance. Despite numerous studies focusing on team creative performance, few have examined team creative performance in scientific research teams. We identified the roles of benevolent leadership and creative self-efficacy in facilitating team creative performance, which helped us develop a comprehensive understanding of the attributes of team leaders and individual cognitive processes that promote team creative performance. Specifically, these results revealed that benevolent leadership was positively related to creative self-efficacy, which ultimately boosted team creative performance.

The article "Benevolent Leadership and Team Creative Performance: Creative Self-Efficacy and Openness to Experience" was published in 2022. Journal: Front Psychol.

Second, this study has theoretical implications for the benevolent leadership literature. Despite previous studies supporting the positive effect of such leadership on team creative performance, the literature focusing on the underlying mediating mechanism is limited. Only a few studies identified the team action process (Li et al., 2018), perceived supervisory support (Chan, 2017), and leader–member exchange (Chan and Mak, 2012) as mediators. We enriched these findings by demonstrating that creative self-efficacy mediates the positive effect of benevolent leadership on team creative performance, especially for scientific research teams in Chinese higher educational settings.

Third, this study contributes to the literature on team personality composition. Although past research has revealed that the average level of a team’s personality moderates the relationship between antecedent variables and team performance (Barrick et al., 1998; Zhou, 2003), the influence of variance on team openness to experience has rarely been investigated. Using the supplementary fit perspective, we extend this branch of research on moderators of team personality composition by demonstrating that the team-mean-level of and team variance on openness to experience moderate the relationship between creative self-efficacy and team creative performance.

### Practical Implications

Our findings offer practical implications. Benevolent leaders can promote team performance through providing support, expressing caring and showing concern for team members. Previous research has found that leader benevolence engenders affective trust, positive emotions and perceived support, which prompts team members to repay the perceived benevolence with improved performance (Chen et al., 2014). As benevolent behaviors were beneficial to team creative performance, scientific research team leaders should employ a benevolent leadership style to achieve the best results. What’s more, managers of the organizations should provide adequate resources and trainings to leaders or supervisors to act more benevolently. In addition, benevolent leadership is an important leadership style in the context of higher education; we, therefore, must adopt it. Universities should encourage team supervisors to care for graduate students while providing academic guidance to help graduate students overcome academic problems and achieve excellent academic achievements.

The article "Benevolent Leadership and Team Creative Performance: Creative Self-Efficacy and Openness to Experience" was published in 2022. Journal: Front Psychol.

Second, the importance of creative self-efficacy has been emphasized by many researchers (Tierney and Farmer, 2011; Farmer and Tierney, 2017). According to our findings, benevolent leaders can facilitate team creative performance through creative self-efficacy. Creative self-efficacy provides individuals with the belief that they can achieve their goals, thus, enhancing their persistence for engagement in creative endeavors, broadening their search cope for information, enriching their useful strategies from new perspectives (Bandura, 1977; Tierney and Farmer, 2011), thereby enhancing team creative performance. To promote team creative performance, we recommend that teams or organizations should encourage team member’s creative self-efficacy in order to improve creativity. In scientific research cooperation, team supervisors can assign easy scientific research tasks for graduate students from the beginning and gradually increase the difficulty of scientific research tasks to help graduate students form a positive, creative self-efficacy. Scientific research teams should also encourage knowledge sharing and practical exchanges. They should improve graduate students’ creative efficacy by providing sufficient social and academic support.

Furthermore, our findings suggest that the team personality composition of openness to experience could influence the degree to which creative self-efficacy affects team creative performance. For creative self-efficacy to be positive and improve team creative performance, we propose that team leaders or managers who interested in promoting team creative performance will find it advantageous to take team members’ personalities into consideration, and create the context that with a high average level and low variance on openness to experience. Team leaders should evaluate personality in team member selection and staffing, with consideration given to the person-environment fit theory, so that members can complement each other. In the context of higher education, although team supervisors should guide graduate students to “teach without distinction” from the perspective of educational concepts. We still suggest that team supervisors take graduate students’ personality traits as a reference for recruiting students when building scientific research teams. The team-mean-level or the team variance on openness to experience will regulate team creative performance.

The article "Benevolent Leadership and Team Creative Performance: Creative Self-Efficacy and Openness to Experience" was published in 2022. Journal: Front Psychol.

### Limitations and Future Direction

Our study has several limitations to consider. First, to avoid common method bias, we utilized team leader ratings of team creative performance and measured the antecedent, mediator, moderator, and outcome at two different time points. Although this study found no serious common method bias, problems still exist in using subjective evaluation to measure team creative performance. In the future, researchers can take scientific research teams of specific disciplines as the research sample and adopt objective indicators to measure the creative performance of scientific research teams. What’s more, future studies could collect data apart from self-report measures, such as by adopting an experimental design to validate the causal effect of benevolent leadership on team creative performance, the mediating effect of creative self-efficacy, and the moderating effect of team personality composition.

Second, the cross-sectional data used in this study cannot make a rigorous judgment on the causal relationship between research variables. Hence, reflecting on the dynamic influence process of benevolent leadership, creative self-efficacy, openness to experience, and team creative performance isn’t easy. Future research can adopt a longitudinal tracking method to further explore the mechanism of the relationship between benevolent leadership and team creative performance.

Third, this study only analyzed the data from a single level, ignoring the impact of individual and organizational factors on the team creative performance. Future studies could include variables at the individual and organizational level, and adopt multi-level analysis to investigate the possible influence of individual and organizational factors on the mechanism of team creative performance comprehensively. In addition, our findings suggested that creative self-efficacy was a partial mediator, indicating that there may be other mediating factors that remain to be explored. To extend the benevolent leadership theory, future studies should explore relevant variables (such as communication, cooperation, and knowledge sharing) that may mediate the relationships studied herein.

Finally, the questionnaires were distributed in Chinese universities, and the team members were postgraduates in universities in one province, which may weaken the generalizability of the results. For example, Chinese people tend to interpret perceived benevolence as a sign of a personalized leader-subordinate relationship, which is guided by mutuality and reciprocity (Farh and Cheng, 2000). Therefore, although benevolent leadership has been found to be beneficial to team creative performance, this positive relationship may not be representative of different contexts or individualistic cultures. Future research should further examine the effects of benevolent leadership on outcomes. What’s more, benevolent leadership belongs to a dimension of paternalistic leadership. Still, a person can also have the other two paternalistic leadership styles at the same time (authoritarian and moral leadership). These three kinds of paternalistic leadership can produce the main effect independently and possibly have complex effects on team creative performance through different combinations. Thus, future research can explore the combined impact of paternalistic leadership on team creative performance.

The article "Benevolent Leadership and Team Creative Performance: Creative Self-Efficacy and Openness to Experience" was published in 2022. Journal: Front Psychol.

## Conclusion

The finding that the contingent effects of team personality composition of openness to experience influence the effect of benevolent leadership on team creative performance through creative self-efficacy promotes our understanding of cognitive processes and team performance. Effectiveness of research teams requires benevolent leadership, creative self-efficacy, and a high average team level of or a low level of variance on openness to experience. This information could be valuable to team leaders in managing their teams better.

## Data Availability Statement

All datasets presented in this study are included in the article/Supplementary Material.

## Ethics Statement

The studies involving human participants were reviewed and approved by Academic Ethical Group of The Faculty of Education, Soochow University. The patients/participants provided their written informed consent to participate in this study.

## Author Contributions

ZX and FY developed the research design. HY was responsible for the data collection as well as for the application of analytical tools. FY and ZX were responsible for article editing. All authors listed have made a substantial, direct, and intellectual contribution to the work and approved it for publication.

## Conflict of Interest

The authors declare that the research was conducted in the absence of any commercial or financial relationships that could be construed as a potential conflict of interest. The reviewer JD declared a shared affiliation with two of the authors HY and FY to the handling editor at time of review.

## Publisher’s Note

All claims expressed in this article are solely those of the authors and do not necessarily represent those of their affiliated organizations, or those of the publisher, the editors and the reviewers. Any product that may be evaluated in this article, or claim that may be made by its manufacturer, is not guaranteed or endorsed by the publisher.
